# OsPIE1, the Rice Ortholog of Arabidopsis PHOTOPERIOD-INDEPENDENT EARLY FLOWERING1, Is Essential for Embryo Development

This article has been retracted.

**DOI:** 10.1371/journal.pone.0011299

**Published:** 2010-06-24

**Authors:** Yonghan Xu, Minjuan Deng, Jianfei Peng, Zhanghua Hu, Lieming Bao, Junming Wang, Zhi-Liang Zheng

**Affiliations:** 1 Province Key Laboratory of Genetic Engineering on Plant Metabolism, Virology and Biotechnology Institute, Zhejiang Academy of Agricultural Sciences, Hangzhou, China; 2 College of Biosafety Science and Technology, Hunan Agricultural University, Changsha, China; 3 Crop Science and Nuclear Utilization Institute, Zhejiang Academy of Agricultural Sciences, Hangzhou, China; 4 Department of Biological Sciences, Lehman College, City University of New York, Bronx, New York, United States of America; University of Massachusetts Amherst, United States of America

## Abstract

**Background:**

The SWR1 complex is important for the deposition of histone variant H2A.Z into chromatin necessary to robustly regulate gene expression during growth and development. In *Arabidopsis thaliana*, the catalytic subunit of the SWR1-like complex, encoded by *PIE1* (*PHOTOPERIOD-INDEPENDENT EARLY FLOWERING1*), has been shown to function in multiple developmental processes including flowering time pathways and petal number regulation. However, the function of the *PIE1* orthologs in monocots remains unknown.

**Methodology/Findings:**

We report the identification of the rice (*Oryza sativa*) ortholog, *OsPIE1*. Although *OsPIE1* does not exhibit a conserved exon/intron structure as Arabidopsis *PIE1*, its encoded protein is highly similar to PIE1, sharing 53.9% amino acid sequence identity. *OsPIE1* also has a very similar expression pattern as *PIE1*. Furthermore, transgenic expression of *OsPIE1* completely rescued both early flowering and extra petal number phenotypes of the Arabidopsis *pie1-2* mutant. However, homozygous T-DNA insertional mutants of *OsPIE1* in rice were embryonically lethal, in contrast to the viable mutants in the orthologous genes for yeast, *Drosophila* and Arabidopsis (*Swr1*, *DOMINO* and *PIE1*, respectively).

**Conclusions/Significance:**

Taken together, our results suggest that OsPIE1 is the rice ortholog of Arabidopsis PIE1 and plays an essential role in rice embryo development.

## Introduction

Chromatin remodeling is a dynamic process that controls eukaryotic gene expression critical for various developmental events. Chromatin remodeling involves histone modifications, histone variant deposition and DNA methylation. While the canonical histones are deposited into chromatin strictly during the S phase of cell cycle, histone variants can be incorporated into chromatin during the entire cell cycle. Therefore, histone variants are involved in specialized cellular functions.

Among the currently identified families of the core histones H2A, H2B and H3, the H2A family of histone variants has the largest number of variants (reviewed in [1], [2]). H2A variants include MacroH2A (which is involved in mammalian X chromosome inactivation), H2A.X (important for DNA repair), and the most evolutionary conserved variant H2A.Z (involved in transcriptional control). H2A.Z has been characterized in various species including yeast, animals and plants. While H2A.Z is encoded by single gene in yeast, *Drosophila* and human, the Arabidopsis genome likely contains four genes (*HTA4*, *HTA8*, *HTA9* and *HTA11*) that encode different members of H2A.Z [1], [3], [4]. Knockdown transgenic plants of *HTA8*, *HT9* and *HTA11* individually or all three genes together are viable [4], [5], [6]. So far it has not been determine whether H2A.Z is essential for Arabidopsis development through analysis of knockout mutants. In other kingdoms, H2A.Z has been shown not to be essential in yeast, but mutations in H2A.Z lead to lethality in *Tetrahymena* [7], *Drosophila* [8], and *mouse* [9]. Furthermore, although the essential function of H2A.Z remains to be investigated, it has been suggested that H2A.Z plays a critical role in either transcriptional repression or activation by occupying the promoter regions of chromatin [2], [10]. Most recently, Arabidopsis H2A.Z has been shown to protect genes from DNA methylation [11].

The deposition of H2A.Z variants to chromatin is catalyzed by the ATP-dependent SWR1 complex in yeast, dTIP60 complex in *Drosophila*, SRCAP and TRRAP/TIP60 complexes in humans, or SWR1-like complex in Arabidopsis [12], [13] [4], [5], [14]. The catalytic subunit of these complexes is Swr1 in yeast [12], [15], Domino in *Drosophila* [13], [16], SRCAP in humans [17], [18], and PHOTOPERIOD-INDEPENDENT EARLY FLOWERING 1 (PIE1) in Arabidopsis [4], [5], [19]. These proteins contain an ATPase domain and belong to the SNF2 family of chromatin remodeling factors. This type of complex also contains other subunits, for example, up to 13 in yeast. Genetic studies reveal that several subunits, Act1, Arp4, Swc4, Rvb1 and Rvb2, are essential for cell viability, while other subunits are not [1], [20], [21].

In Arabidopsis, orthologs for all subunits, except for the two yeast subunits (Swc3 and Swc7), have been identified [1]. However, only a few of them have been functionally characterized. These include PIE1, ARP6/SUF3/ESD1, and SEF/SWC6 [5], [19], [22], [23], [24], [25], [26]. Analysis of mutants of these genes revealed pleiotropic developmental phenotypes, such as changes in plant stature, leaf shape and size, flowers with extra petals, and early flowering under both long- and short-day photoperiods. Furthermore, the early flowering and leaf serration phenotype can also be observed in Arabidopsis H2A.Z knockdown transgenic plants [4], [5], demonstrating a consistent function for the H2A.Z variant and its regulatory SWR1-like complex. Among these phenotypes, flowering time has received the most attention. Several studies have demonstrated that this complex regulates the deposition of H2A.Z variant into chromatin at the *FLOWERING LOCUS C* (*FLC*) locus and consequently exerts the transcriptional control of *FLC*, a MADS box transcription factor that acts as a critical floral repressor of flowering [4], [5], [19], [23], [25]. Arabidopsis is a facultative long-day plant, and for the winter-annual ecotype, vernalization can de-repress *FLC*, which in turn activates the expression of several flowering time-related genes, such as *FT* and *SOC1*, leading to elevated expression of *AP1* and *LEAFY* genes and ultimately flowering [27], [28].

Rice is an economically important crop. Preliminary phylogenetic analyses indicate that the rice genome contains three genes coding for H2A.Z variants, and one ortholog of ARP4 and ARP6 respectively [4], [23]. Except for this information, virtually very little is known regarding the components of the SWR1-like complex and their functions in rice and indeed any other monocot species. As a first step towards dissecting the SWR1-like complex and its function in rice growth and development, we attempted to identify the Arabidopsis PIE1 ortholog (OsPIE1). Surprisingly, homozygous T-DNA insertional mutants of *OsPIE1* are embryonically lethal. This suggests that unlike the catalytic subunit of the SWR1 complex in Arabidopsis, yeast and animals, OsPIE1 plays an essential role in rice embryo development.

## Results

### Identification of the *OsPIE1* Gene in Rice

To identify the rice ortholog of PIE1, we used the Arabidopsis PIE1 protein (Accession number: AY279398) encoded by AT3G12810 [19] to perform a BLAST search in the rice genome database (http://signal.salk.edu/cgi-bin/RiceGE). This search resulted in one rice genomic sequence (Os02g46450) and one cDNA clone (AK120785, clone name: J023010H23, with the length of only 3,375 bp). Apparently, this cDNA clone only represents a partial *OsPIE1* cDNA encoding the carboxyl-terminus. Therefore, we used RT-PCR to amplify the full-length cDNA. Using both 5′ and 3′ fragments of OsPIE1 cDNA as the mixed probes in Northern blot, we detected a single, strongly hybridized band (data not shown) of 6.7 kb in size, consistent with its predicted length. This indicates that *OsPIE1* is likely a single copy gene, encoded by Os02g46450 and located in the upstream of chromosome 2. The *OsPIE1* cDNA molecule was sequenced and the sequence has been deposited into the NCBI GenBank with an accession number GQ906768. Sequencing results revealed that there is an additional exon between the predicted ninth and tenth exons (Figure 1A). In addition, we also found that *OsPIE1* has a very different genomic structure, with 23 exons and 22 introns, compared to *PIE1* which contains 20 exons and 19 introns (Figure 1A).

**Figure 1:** Genomic structure of *OsPIE1* gene and sequence alignment of OsPIE1 homologs. (**A**) Genomic structure of *OsPIE1* and Arabidopsis *PIE1* genes. The translation start and stop sites are indicated. Exons are presented as filled black rectangles, and introns or intergenic sequences are presented as solid lines. For *OsPIE1*, the upper diagram (“predicted”) depicts the predicted structure of the *OsPIE1* gene in the RiceGE database with 21 introns and 22 exons. The lower diagram (“cloned”) represents the structure of the *OsPIE1* gene cloned and verified in this study, with an extra exon within the predicted 9th intron, corresponding to nucleotides 2368 to 2437 of the genomic fragment. (**B**) Domains of *OsPIE1*. Domains are predicted by the SMART program (http://smart.embl-heidelberg.de) and the amino acid numbers of these domains are indicated. The two putative bipartite nuclear localization signals (NLS) at the N-terminal and C-terminal regions of OsPIE1 are KRQKTLEAPKEPRRPKT and KKRDLIVDTDEE KTSKK, respectively. (**C**) Sequence alignment of the SNF_N domains of OsPIE1, Arabidopsis PIE1, *Drosophila* DOMINO A, human SRCAP, and yeast SWR1. Numbers indicate the amino acid positions. (**D**) Sequence alignment of HELICc domain. Amino acids corresponding to the domain are underlined. Numbers indicate the amino acid positions. (**E**) A phylogenetic tree of *OsPIE1* orthologs from several organisms. The names of organisms are indicated in parenthesis, and bootstrap values are provided for the indication of reliability for each node.

### Comparative Analysis of the Predicted OsPIE1 Protein and Other PIE1 Homologues

Based on the expressed *OsPIE1* cDNA sequence we have obtained, OsPIE1 protein, like Arabidopsis PIE1, has an HAS domain at the N-terminus, two domains highly similar to the SNF2_N and HELICc domains, and a SANT domain in the C-terminus (Figure 1B). Two bipartite nuclear localization signals (NLS) are also present (Figure 1B), indicating that both OsPIE1 and PIE1 are likely localized to the nucleus [4], [19]. The SNF2_N and HELICc domains are present in the SWI2/SNF2 and ISWI class of chromatin remodeling proteins, which are involved in the transcriptional activation or repression of target genes. For these two domains, OsPIE1 and PIE1 share high similarity with DOMINO (Accession number: AF076776) from *Drosophila* [16], SRCAP (Accession number: AF143946) from human [17], and SWR1 (Accession number: NP_010621) from yeast [15], with amino acid identity ranging from 58 to 77% (Figure 1, C and D).

A C-terminal region of OsPIE1 also exhibits similarity to the SANT domain (Figure S1). The SANT domain was found originally in SWI3, ADA2, N-CoR, TFIIIB B and ISWI, and it is characteristic of the ISWI family members [29]. Furthermore, it has been shown that the N-terminal half of the SANT domain is required for interactions with histone acetyltransferases or histone deacetylases, while the C-terminal half is required for the interaction with chromatin [30], [31], [32]. Although the amino acid identity of the SANT domains between PIE1 and other proteins, including DOMINO [16], SRCAP [17], and SWR1 from yeast [15], is very low, we found that the conserved and functionally important residues of the SANT domain are still present in this region for the PIE1 orthologs (Figure S1; see also [19]). Additionally, like PIE1, OsPIE1 has a unique 11-amino acid linker, GGAF(AGGA for PIE1) YRGRYRHP), between the N-terminal and C-terminal halves of the SANT domain (Figure S1). This linker is absent in DOMINO, SRCAP and SWR1.

Of particular note, except for the domains described above, other regions of OsPIE1 and PIE1 are quite divergent from the proteins of the SWI2/SNF2 and ISWI family in non-plant species (data not shown). In contrast, OsPIE1 and PIE1, which are from dicotyledon and monocotyledon model plants rice and *Arabidopsis*, respectively, exhibit a similarity as high as 53.9% at the amino acid level for the full-length proteins (Figure S1). They are almost identical to each other (up to 95% identity) in all of the important functional domains as described above (Figure 1, C and D; Figure S1). Together with phylogenetic analysis using yeast Swr1 and its orthologs in Arabidopsis, rice, human and *Drosphila* (Figure 1E), these results suggest that OsPIE1 protein is more closely related to Arabidopsis PIE1 than to any other homologues from human, yeast, and *Drosophila*.

### *OsPIE1* Exhibits a Similar Expression Pattern as Arabidopsis *PIE1*

The highly similar amino acid sequences for rice and Arabidopsis PIE1 proteins led us to hypothesize that *OsPIE1* has a similar expression pattern as *PIE1*. To investigate the temporal and spatial expression patterns of *OsPIE1*, we used both promoter∶reporter assay and reverse transcriptase (RT)-PCR analysis. To analyze *OsPIE1* promoter activity, a 1.6 kb genomic fragment upstream of the ATG start codon was used to drive the β-glucuronidase (GUS) reporter expression. A total of 16 independently transformed rice lines were obtained and most of these lines showed similar GUS staining patterns. We observed that GUS activity was detected in all rice plant tissues or organs tested, with a higher expression in the shoot apical meristem, root, young shoot, panicle and spikelet (Figure 2).,High *OsPIE1*:*GUS* expression was detected in the divisional and young panicles just prior to heading (Figure 2A). During the heading stage, the highest *OsPIE1*:*GUS* expression was detected in the flowering spikelets and the divisional zone (Figure 2 B–E). GUS activity was also present in the mature seed (Figure 2C), but almost absent in the leaf (Figure 2D).

**Figure 2:** Expression patterns of *OsPIE1* in rice. (**A**) to (**F**) Histochemical GUS assays in the *OsPIE1* promoter:GUS transgenic lines. (**A**) GUS staining in the primary root with lateral roots. Arrow indicates the lateral root initiation site. (**B**) to (**E**) GUS staining in young spikelets (**B**), the mature spikelet (**C**), the young leaf (**D**) and the flower (**E**). (**F**) GUS activity in the young shoot (a), including the rapid elongation zones of culm internodes before panicle development (see the enlarged images, b and c), and the elongation zone of peduncle (d). (**G**) RT-PCR analysis of *OsPIE1* mRNA expression in different tissues or organs. Tissues or organs used were: Ca, callus; R,7-day-old roots; SL,7-day-old leaves; ML, mature leaves; FLB, flag leaf blade; FLS, flag leaf sheath; St, stem; P1,1 to 2-cm-long panicles; P2, 3 to 5-cm-long panicles; and P3, 5 to 8-cm-long panicles. The rice *Actin* gene was used as an internal control.

RT-PCR analysis using RNA extracted from various tissues and organs showed that *OsPIE1* is expressed in the growing roots, stems, flowers and preferentially in the shoot apical meristem and the spikelet (Figure 2G). *OsPIE1* is also expressed in flag leaf blade and sheath, but at very low level in mature leaves. Furthermore, at the heading stage, flowering panicles and stems accumulated the *OsPIE1* transcript at the highest level, followed by panicles before flowering. This result is largely consistent with the promoter:GUS expression patterns (Figure 2, A–F), indicating that the 1.6 kb promoter fragment likely contains all of necessary *cis*-elements for proper expression of *OsPIE1*. The preferential expression of *OsPIE1* in floral organs compared to leaves is very similar to that of *PIE1* in Arabidopsis [19].

### Transgenic Expression of *OsPIE1* Rescues the Early Flowering Phenotype in the *Arabidopsis pie1* Mutant

The highly similar protein sequences and expression patterns between *OsPIE1* and *PIE1* led us to hypothesize that OsPIE1 also has similar functions as PIE1 in the control of flowering time and petal number. To test this hypothesis, we constructed the Arabidopsis *PIE1* promoter:*OsPIE1* cDNA expression cassette and investigated whether expression of *OsPIE1* could functionally complement the early flowering and iregular petal number phenotype in transgenic plants of Arabidopsis *pie1-2*, a likely null allele [19]. Among 50 T1 plants, 26 flowered later than *pie1-2* and close to wild-type Col. The seeds from these T1 plants were then tested for the segregation of hygromycin resistant versus sensitive seedlings, and we found that 20 lines exhibited 3∶1 segregation ratios. These 20 lines, each with a single T-DNA insertion, were shown to co-segregate the presence of transgene with normal flowering time phenotype (data not shown). As shown in Fig. 3A, two representative lines of transgenic *pie1-2* plants did not flower, similar to Col but in sharp contrast to *pie1-2* which already flowered. Quantitative analysis of flowering time showed that indeed the transgenic lines had similar number of rosette leaves from seed germination to flowering as Col, under both long-day and short day conditions (Table 1). Furthermore, they also reverted the abnormal petal number (three, five or six) to normally four petals (Figure 3, B–F).

**Figure 3:** Rescue of the *pie1-2* mutant phenotypes by transgenic expression of *OsPIE1*. (**A**) to (**F**) Phenotypes of transgenic *Arabidopsis pie1-2* plants transformed with *OsPIE1* under the control of the Arabidopsis *PIE1* promoter. (**A**) Plants of two representative transformant (middle), WT (left) and the *pie1-2* mutant (right) grown under long-day conditions (16 h light/8 h dark) until *pie1-2* plants flowered. Inflorescence of transgenic *pie1-2* plant (**C**) was compared with that of WT (**B**) and *pie1-2* mutant (**E**). Abnormal floral organ number (with an extra petal indicated by arrowhead in **F**) in *pie1-2* mutant was rescued in transformants of *pie1-2* (with 4 petals; **D**). (**G**) RT-PCR analysis of *PIE1* and *OsPIE1* expression patterns. Expression of *PIE1* was conducted in Col (wild-type), and *OsPIE1* in *pie1-2* transformants (Arabidopsis *PIE1* promoter:*OsPIE1* cDNA). Tissues or organs were collected from adult plants grown in long days. Arabidopsis *ACT2* was used as an internal control. (**H**) Gel blot analysis of *FLC* expression in various tissues or organs from *pie1-2* or one representative *pie1-2* transformant (transformed with *OsPIE1* under the control of Arabidopsis *PIE1* promoter). The blots were probed first with *FLC* and then re-probed with Arabidopsis *UBQ10* as an internal control.

**Table 1:** Rosette leaf number of *pie1-2* and *pie1-2* transformants at flowering in long and short days.

Light Conditions	Wild-type	*pie1-2* Transformants	*pie1-2*
Long days	9.7±1.4	9.4±0.6	6.8±0.5
Short days	40.9±4.9	42.3±3.	17.3±1.5

Values shown are mean rosette leaves numbers±SD at flowering. At least 15 plants were scored for each genotype and treatment.

To confirm that the phenotypic rescue of *pie1-2* is the result of proper expression of *OsPIE1*, RT-PCR analysis was performed. Results showed that expression of *OsPIE1* driven by the Arabidopsis native *PIE1* promoter was very high in seedlings and flowers but barely detectable in leaves (Figure 3G, lower panel). This pattern was quite similar to *PIE1* expression in Col (Figure 3G, upper panel; also see [19]), except that transgenic *OsPIE1* expression was also high in roots compared to relatively weak expression of *PIE1* in Arabidopsis roots.

Because it has been demonstrated that the early flowering phenotype in *pie1* mutants is mainly due to the reduced expression of *FLC* [19], we decided to assess whether native *FLC* expression is restored in *OsPIE1* expressing transgenic lines of *pie1-2*. Results from Northern blot using *FLC* as a probe showed that in contrast to weak expression of *FLC* in *pie1-2*, transgenic expression of *OsPIE1* under the control of *PIE1* promoter induced the strong *FLC* expression in the shoot apex but not in other organs tested (Figure 3H). Taken together, we have demonstrated that OsPIE1 can functionally replace PIE1 in the control of flowering time and petal number in Arabidopsis. This suggests that the biochemical function of OsPIE1 and PIE1 are evolutionally conserved [4], [5], [19].

### Homozygous *Ospie1* T-DNA Insertion Mutants Are Embryonically Lethal

To test whether *OsPIE1* may also function in the control of flowering time and petal number regulation in rice, T-DNA knockout mutants of *OsPIE1* were isolated and characterized Two independent alleles, *Ospie1-1* and *Ospie1-2* (corresponding to the PFG_3A-60036 and PFG_1B-21620 stocks, respectively), were obtained from the rice T-DNA insertion mutagenesis collection at the Plant Functional Genomics Laboratory [33]. Both mutants have a T-DNA insertion in the 11th (926 nucleotides downstream of ATG in genomic DNA) and 12th (964 nucleotides downstream of ATG) introns, respectively. The T-DNA insertion sites in *OsPIE1* suggest that *Ospie1-1* and *Ospie1-2* may cause loss of *OsPIE1* function. Using PCR- based genotyping of T-DNA insertions in at least 300 segregating plants derived from self-pollinated heterozygous plants (*Ospie1-1/+* and *Ospie1-2/+*), we failed to obtain any homozygous plants for both alleles and thus we were unable to determine whether the mutations are null or leaky. Nevertheless, we found that the progeny from self-fertilized *Ospie1-1*/+ or *Ospie1-2*/+ parental plants exhibited a segregation ratio of 2∶1 for heterozygotes and WT plants (Table 2). This genetic analysis indicates that the homozygous T-DNA insertion mutants in *OsPIE1* are likely lethal. No obvious phenotype was observed in all of heterozygous plants. However, when the seeds collected from the self-pollinated *Ospie1-1*/+ and *Ospie1-2*/+ plants were examined, 21–25% of the seeds were empty (indicated by red arrowheads in Figure 4A and shown in Figure 4B), as compared to WT which had 95% of plump yellowish (filled) seeds (Figure 4C). The percentage of filled grains is consistent with the expected 3∶1 ratio of plump yellowish seeds versus empty seeds for the progeny from self-pollinated *Ospie1-1*/+ or *Ospie1-2*/+ plants. Together with the genotyping result, our data suggest that all of the homozygous recessive (*Ospie1-1* and *Ospie1-2*) embryos are inviable.

**Figure 4:** Phenotypic characterization of *Ospie1* mutants. (**A**) Spikelets of self-pollinated wild-type (WT), *Ospie1-1*/+, and *Ospie1*-2/+. Red arrowheads indicate the panicels of abnormal empty seeds for each of the three genotypes. (**B**) Representative images of normal WT seeds and empty seeds from self-pollinated *Ospie1-1/+* and *Ospie1-2/+* plants. Half of the husk was removed for visualizing endosperms. No endosperm developed normally in those empty seeds of *Ospie1-1/+* and *Ospie1-2/+* plants. (**C**) Quantitative analysis of grain setting rates for heterozygous *Ospie1* plants. Grain setting rate is the percent of filled grains over the sum of filled and empty grains for each plant. Data shown are means ± SD of 30 plants for each genotype. The experiment was repeated three times, with a similar result.

**Table 2:** Segregation of T-DNA in *Ospie1* heterozygous mutants.

Genotypes of Self-pollinated Plants	Progeny with One T-DNA Insertion	Progeny with No T-DNA Insertion	*X* ^2^-test Result
*Ospie1-1*/+	203	97	*X* ^2^-value = 0.135 (*p*-value>0.05)
*Ospie1-2*/+	212	98	*X* ^2^-value = 0.413 (*p*-value>0.05)

PCR-based genotyping was performed in the progeny from self-pollinated parental plants. *X* ^2^-test was performed to show whether it is consistent with a 2∶1 segregation.

To determine whether the homozygous lethality is due to the defects in gametes or embryos, reciprocal crosses were performed between WT and *Ospie1-1/+*, and between WT *Ospie1-2/+*. Due to the abnormal high temperatures in the growing field in tropical Hainan province in China in 2010, the grain setting ratios for the F1 progeny derived from all types of crosses were unexpectedly low (approximately 10%), which were similar to the control cross, WT×WT (Table 3). However, we found no statistical difference in the setting ratios for the F1 progeny derived from the reciprocal crosses involving WT and *Ospie1-1* or WT and *Ospie1-2*. Furthermore, PCR genotyping of those F1 progeny derived from individual crosses showed consistent 1∶1 segregation ratios for *Ospie1* heterozygotes and WT in all of the reciprocal crosses (Table 3). These results support the idea that gametes are unaffected by *Ospie1-1* and *Ospie1-2* mutations and that the homozygous lethality of *Ospie1* mutants is likely caused by a defect in embryo development. Indeed, we observed that 10 days after self-pollination, the embryos in the abnormally developed grains from *Ospie1-1/+* or *Ospie1-2/+* were very small, compared to the normal WT embryos (Figure 5). Those grains with smaller embryos showed endosperm shrinkage (Figure 5), which became empty seeds when mature (Figure 4B).

**Figure 5:** Abnormal embryos in *Ospie1* mutants. Upper panels show the representative seeds (with the hull completely removed) in wild-type (WT) and the abnormally developed grains in self-pollinated *Ospie1-1/+* and *Ospie1-2/+* plants, respectively. The white rectangular box indicates the approximate position of embryo. The bar represents 1.99 mm for all three images in the upper panels. Lower panels show the embryos collected from the seeds indicated in the upper panels, with the bar representing 0.1 mm.

**Table 3:** Reciprocal crosses between Ospie1 hetrozygotes and wild-type.

Type of Crosses (male × female)	Setting Rate (%)	Number of *Ospie1* Heterozygotes in F1	Number of Wild-type in F1	*X* ^2^-test Result
*Ospie1-1/+* × WT	6.1±1.8	41	43	*X* ^2^-value = 0.048 (*p*-value>0.05)
*Ospie1-2/+* × WT	9.2±4.6	31	34	*X* ^2^-value = 0.138 (*p*-value>0.05)
WT × *Ospie1-1/+*	10.1±4.8	31	32	*X* ^2^-value = 0.016 (*p*-value>0.05)
WT × *Ospie1-2/+*	11.0±5.1	19	21	*X* ^2^-value = 0.100 (*p*-value>0.05)
WT × WT	10.8±4.7	0	93	*X* ^2^-value = 93.000 (*p*-value<0.05)

Reciprocal crosses between wild-type and *Ospie1-1* or *Ospie1-2* heterozygous plants were performed and the setting rates for each cross were scored. Data represented the average ±SD for 5–8 plants in each cross. No statistical significant difference was observed in setting rates between these genotypes. Those filled grains in F1 were then PCR genotyped to determine the number of *Ospie1* heterozygotes and wild-type. *X^2^*-test was used to determine that they followed the 1∶1 segregation ratio. A cross involving wild-type (WT) was also performed as a control.

## Discussion

Several lines of evidence together demonstrate that OsPIE*1*, encoded by Os02g46450, is the true rice ortholog of Arabidopsis PIE1. First, at the amino acid sequence level, these two proteins share 53.9% identity. Second, protein domain prediction and comparison reveal that OsPIE1 is very similar to PIE1, with almost identical domains. Third, phylogenetic analysis also places OsPIE1 as the most closely related protein of PIE1, compared to other catalytic subunits in yeast and animals. Fourth, *OsPIE1* exhibits a very similar tissue and developmental expression pattern as *PIE1*. Fifth and importantly, transgenic expression of *OsPIE1* in Arabidopsis *pie1-2* mutant complements the *pie1-2* phenotypes with regard to flowering time and petal number. Therefore, the identification of OsPIE1 as the ortholog of the catalytic subunit of the SWR1-like complex in rice provides the basis to dissect the physiological function of OsPIE1 in the future.

We were surprised to observe that homozygous T-DNA insertions lead to lethality in rice. Lethality could be caused by the failure or defects at any stage of reproductive development, such as reduced fertility of male and female gametes, failure of fertilization, or more likely abortion of embryo development. However, we have observed that pollen grains collected from both *Ospie1-1/+* and *Ospie1-2/+* plants are viable, as indicated by similar kalium iodide staining as WT pollen grains (data not shown). Furthermore, when reciprocal crosses were performed between WT and heterozygous *Ospie1-1* or *Ospie1-2* mutants, they showed similar F1 setting ratios, and genotyping of the F1 progeny confirmed the 1∶1 segregation ratio for heterozygotes and WT. In addition, we also observed that young embryos (10 days after pollination) in the abnormal grains derived from the self-pollinated *Ospie1-1* and *Ospie1-2* heterozygous plants were much smaller than the embryos in the normal grains of WT plants. Therefore, homozygous lethality in the T-DNA insertional mutants of *OsPIE1* is caused by the abortion of embryos. This demonstrates an essential role for OsPIE1 in proper rice embryo development.

The essential function for OsPIE1 in rice embryo development is a novel finding. Some studies have demonstrated the importance of histone variants in mammalian reproduction (reviewed in [34]). For example, H2A.Z is essential for embryo development in *Drosophila* and mouse [8], [9]. In addition, the H2A.F/Z variant hv1 has also been shown to be essential in the ciliated protozoan, *Tetrahymena thermophila* [7]. However, loss-of-function mutants for the genes encoding the components of the SWR1-like complexes are viable in these organisms. Interestingly, although H2A.Z is not essential in yeast, the H2A.Z mutation is synthetically lethal with an H4 histone mutation [35]. Furthermore, five subunits of the SWR1 complex, Act1, Arp4, Swc4, Rvb1 and Rvb2, play an essential role in yeast cell viability [1], [20], [21]. In Arabidopsis, the mutants or knockdown transgenic plants for the genes encoding H2A.Z variants and the three components of the SWR1-like complex (PIE1, ARP6, SEF) exhibit an obvious early flowering phenotype and the subtle phenotypes in leaf morphology and petal number [4], [5], [6], [19], [22], [23], [24], [25], [26]. The lethal phenotype has not been reported, although the *arp6* mutant of Arabidopsis has been shown to reduce female fertility and consequently reduce number of seeds in the silique [23]. Therefore, our finding that the catalytic subunit of the SWR1-like complex can also play an essential role in development is novel. One of the likely explanations for the essential function is that OsPIE1 targets the rice H2A.Z to chromatin at the locus or loci that contain the genes essential for embryo development. Generating *OsPIE1* knockdown transgenic rice plants in the future will, if they are not lethal, help us to determine which aspect of cell growth and embryo development is controlled by OsPIE1 and whether OsPIE1 has a similar physiological function in the control of flowering time in rice.

In summary, we have shown that OsPIE1 is the rice ortholog of Arabidopsis PIE1, the catalytic subunit of the SWR1-like complex in Arabidopsis. OsPIE1 can functionally replace PIE1 in the control of flowering time and petal development, supporting that PIE1 orthologs are evolutionarily highly conserved. Most interestingly, we have shown that this catalytic subunit in rice is essential for embryo development, which has not been reported in Arabidopsis, yeast and animals. Future work should further reveal whether OsPIE1 also functions in the control of flowering time in rice and how it remodels the chromatin associated with the genes essential for embryo development.

## Materials and Methods

### Plant Materials and Growth Conditions

*Ospie1*/+ T-DNA insertion lines in Dongjin (*Oryza sativa* spp *japonica* cv) back- ground were isolated from the POSTECH rice T-DNA insertion mutant bank (http://signal.salk.edu/cgi-bin/RiceGE). The *Ospie1*/+ plants were propagated vegetatively in the summer in Hangzhou City, China and the winter on Hainan Province (close to South China Sea) under natural conditions. Rice materials were harvested from plants grown in the field.

*Arabidopsis* plants (ecotype Columbia) were grown routinely under controlled environmental conditions (23°C day/18°C night, white fluorescent lamps with a light intensity of 150 mmol m^−2^ sec^−1^, 16 h light/8 h dark, and 65% relative humidity). To isolate T-DNA insertion mutant alleles for Arabidopsis *PIE1* (At3g12810), seeds were obtained from either the SALK Collection (http://signal.salk.edu/; *pie1-2*, which is SALK_003776) or the Syngenta Arabidopsis Insertion Library (http://www.nadii.com/pages/collaborations/).

### Cloning of the *OsPIE1* Gene and Genotyping of the *Ospie1* T-DNA Insertion Mutants

The coding sequence (CDS) of *OsPIE1* which encodes 2045 amino acids was PCR-amplified from reverse-transcribed rice cDNA (Invitrogen, Carlsbad, CA, USA), using the following primers: OsPIE1F1, 5′-ATGGCATCAAAAGGTCCTCGATCAAAG-3′; OsPIE1R1, 5′-TCTGGCATTGAG GAGTTGGATCCTCTTAC-3′. Due to the large size of the *OsPIE1* transcript, we obtained the full-length cDNA of *OsPIE1* by amplifying several fragments. Its 5′ untranslated region (UTR) and 3′ UTR sequence of *OsPIE1* were obtained by the method of 5′ rapid amplification of cDNA end (RACE) and 3′ RACE using the kit provided by TaKaRa (TaKaRa, Kyoto, Japan). Primers for 5′-RACE and 3′-RACE were designed according to the manufacturer's instructions. All of the above PCR products were cloned into pMD18-T vector, according to the manufacturer's instructions (TaKaRa, Kyoto, Japan).

Genotyping of the progeny derived from self-pollinated *Ospie1-1/+* and *Ospie1-2/+* plants or from the reciprocal crosses between WT and *Ospie1-1/+* or *Ospie1-2/+* was performed by PCR using the following primers. For *Ospie1-1*: P1LP, 5′-AGTTGTG TACCAGGGCAAGG-3′; P1RP, 5′-GGATCGGACCGATAGTTCAG-3′; 2717LB, 5′-GAACGGCCACAAGTTCAGCGT-3′. For *Ospie1-2*: P2LP, 5′-TGGACTCT GGGAGAGCTAGG-3′; P2RP, 5′-GAAGGCAGTGGG AAAA ACAG-3′; 2715LB, 5′-CTAGAGTCGAGAATTCAGTACA-3′. The PCR was conducted with an initial step of 94°C incubation for 5 min, followed by 30 cycles of 94°C for 30sec, 56°C for 30 sec, and 72°C for 45 sec.

### *OsPIE1* Expression Vector Construction and Plant Transformation

The primers OsPIE1F1-1 and OsPIE1R1-1 (with the Sal I and Pml I sites incorporated as to the above described primers OsPIE1F1 and OsPIE1R1; OsPIE1F1-1, 5′-GTCGACATGGCATCAAAAGGTCCTCGATCAAAG-3′; OsPIE1R1-1, 5′-CACGTG TCTGGCATTGAGGA GTTGGATCCTCTTAC-3′) were used to amplify the 6.13 kb CDS that contains the entire *OsPIE1* coding region. The PCR product was then inserted into the binary vector pCAMBIA1301 after digestion by Sal I and Pml I, resulting in pPNA109. The 1.5 kb Arabidopsis *PIE1* promoter fragment was amplified as previously described [19] and after digestion with EcoR I and Sal I, it was inserted into pPNA109, upstream of *OsPIE1* CDS, resulting in the *OsPIE1* expression vector pPNA119. The resulting construct was introduced into *Agrobacterium tumefaciens* starin EHA105 and then transformed into *pie1-2* mutant via the floral dip method [36]. Transgenic plants were selected on agar-solidified medium containing 0.65 g/L Peter's Excel 15-5-15 fertilizer and 50 µg/ml hygromycin.

### Promoter:GUS Construct and GUS Activity Assay

A 1.6 kb *OsPIE1* promoter fragment was amplified by PCR using two primers: OsPIE1PF, 5′-GTGTGCTGCAGTGGGTAGAAGGGTAATTGAGAGC-3′ and OsPIE1PR, 5′-CCATGTCTAGACTTTCCGAT ATTTTGTAGAGAACTATCT-3′ , with the Pst I and Xba I (underlined) restriction sites incorporated, respectively. The PCR product was then digested with Pst I and Xba I and cloned into pCAMBIA1301 to replace the CaMV 35S promoter, resulting in the *OsPIE1:GUS* reporter construct. The *OsPIE1:GUS* construct was used to transform Nipponbare (*Oryza sativa* spp japonica cv) via the *Agrobacterium*-mediated method as previously described [37]. Histochemical assay for GUS activity in transgenic plants was performed as described [38].

### Reverse Transcriptase (RT)-PCR Analysis

The Trizol reagent (Invitrogen) was used to extract total RNA from various tissues or organs of rice and *Arabidopsis* plants, according to the manufacturer's instructions. RT-PCR was performed using gene-specific primers. *OsPIE1*: OsPIE1F, 5′-CTGAGCGCAACGAGGAATTGGCTGCt-3′, OsPIE1R, 5′-CCCAGCATGCCT GCAGATTCATGATC-3′; Rice *actin*: actin1F,5′-GTCAATAACTGGGATGACATGGAG-3′, actin1R, 5′-AGCTTCATGTATGCCAGG AGATT-3′; and *PIE1*: PIE1F, 5′-GTCCTGAACTCGATGAGGAT-3′, PIE1R,5′-GCAGGGCAATCTCTTCGACATGAT-3′. PCR was performed with 32 cycles for both *OsPIE1* and *PIE1* and 30 cycles for rice *Actin*.

### RNA Gel Blot Analysis

RNA electrophoresis and subsequent blot and hybridization were performed as described elsewhere [39], [40]. Total RNA of 40 µg was loaded on each lane. Briefly, after hybridization for 20 h at 68°C, the membrane was washed once with 2×SSC plus 0.1% SDS at 68°C for 20min, and then with 13 SSC plus 0.1% SDS at 37°C for 30min. The membrane was exposed to the x-ray film (Kodak, Rochester, NY) at 27°C for 3 to 7 d. The *FLC* cDNA fragment lacking the conserved MADS-domain sequences was labeled with [^32^P]dCTP (China Isotope, Beijing) and used as the probe for *FLC*. The blot was first hybridized with the *FLC* probe and then re-probed with the *UBQ10* probe (a 128 bp fragment of AT4g05320 cDNA). The 128 bp *UBQ10* fragment was PCR-amplified using the following primers: sense primer UBQF (5′-TTCACTTGGTCCTGCGTCTTCGTGGTGGTTTC-3′) and antisense primer UBQR (5′-CATCAGGGATTATACAAGGCCCC-3′).

### Phylogenetic Analysis

Amino acid sequences of PIE1and its related proteins were obtained from the NCBI database. The retrieved *PIE1* homolog sequences were aligned using BioEdit software (http://www.mbio.ncsu.edu/BioEdit/bioedit.html), and neighbor-joining trees were generated using the MEGA version 3.1 software [41], with bootstrap values obtained from 500 replications.

### Microscopic Observation of Embryos

Rice seeds were cut into small pieces (3×3 mm) and fixed with 2.5% glutaraldehyde and 1% osmium tetroxide. After a brief rinse with the phosphate buffer (0.1 M Na_2_HPO_4_ and NaH_2_PO_4_, pH 7.0), the specimens were dehydrated in a series of ethanol solutions and acetone and then embedded in Spurr resin. Semi-ultra thin sections (2–4 µm) were prepared using a glass knife and stained with the methylene blue for examination under the microscope LEICA (Model DM LB2).

## Supporting Information

Figure S1 Aligment of OsPIE1 and Arabidopsis PIE1 protein sequences.
(0.05 MB DOC)
